This article has been retracted.

# Inhibition of Tomato Yellow Leaf Curl Virus (TYLCV) using whey proteins

**DOI:** 10.1186/1743-422X-7-26

**Published:** 2010-02-03

**Authors:** Ashraf M Abdelbacki, Soad H Taha, Mahmoud Z Sitohy, Abdelgawad I Abou Dawood, Mahmoud M Abd-El Hamid, Adel A Rezk

**Affiliations:** 1 Plant Pathology Department, Faculty of Agriculture, Cairo University, Giza 12613, Egypt; 2 Dairy Science Department, Faculty of Agriculture, Cairo University, Giza 12613, Egypt; 3 Biochemistry Department, Faculty of Agriculture, Zagazig University, Zagazig, Egypt; 4 Virus and Mycoplasma Department, Agriculture Research Center, Giza 12619, Egypt

## Abstract

The antiviral activity of native and esterified whey proteins fractions (α-lactalbumin, β-lactoglobulin, and lactoferrin) was studied to inhibit tomato yellow leaf curl virus (TYLCV) on infected tomato plants. Whey proteins fractions and their esterified derivatives were sprayed into TYLCV-infected plants. Samples were collected from infected leaves before treatment, 7 and 15 days after treatment for DNA and molecular hybridization analysis. The most evident inhibition of virus replication was observed after 7 and 15 days using α-lactoferrin and α-lactalbumin, respectively. Native and esterified lactoferrin showed complete inhibition after 7 days. On the other hand, native β-lactoglobulin showed inhibition after 7 and 15 days whereas esterified β-lactoglobulin was comparatively more effective after 7 days. The relative amount of viral DNA was less affected by the esterified α-lactalbumin whereas native α-lactalbumin inhibited virus replication completely after 15 days. These results indicate that native or modified whey proteins fractions can be used for controlling the TYLCV-infected plants.

## Introduction

Tomato yellow leaf curl virus (TYLCV) is one of the major and serious diseases of tomato which causes considerable amount of yield loss in Egypt [1-3]. One hundred twenty five million tons of tomatoes were produced in the world in 2007. China, the largest producer, accounted for about one quarter of the global output, followed by the United States, Turkey, India and Egypt. http://www.fas.usda.gov/htp/2009%20Tomato%20Article.pdf. Losses from plant diseases can have a significant economic impact, causing a reduction in income for crop producers, distributors, and higher prices for consumers.

In order to control TYLC-disease, it was found that frequent spray (at 7 days interval) of insecticide, like Cypermethrin (0.01%) or Dimethoate (0.1%) is effective to minimize the disease by controlling its vector whitefly (*Bemisia tabaci*) [4,5].

Researches focused on the use of alternative method to avoid the undesirable effects of the insecticides. In 1940s several investigators suggested the use of milk as spraying or dipping of seedlings for reducing the incidence of virus infections. Recent studies demonstrated the effectiveness of milk in reducing infection of tobacco mosaic virus (TMV) in pepper, tomato, and tobacco [6,7].

Whey represents a rich and heterogeneous mixture of secreted proteins with wide ranging nutritional, biological and food functional attributes. The main constituents of whey are α-lactalbumin (ALA), β-lactoglobulin (BLG) and two small globular proteins that account for approximately 70-80% of total whey protein. Historically, whey has been considered a waste product and disposed of in the most cost-effective manner, or processed into relatively low value commodities such as whey powder and various grades of whey protein concentrate/isolate (WPC, WPI). Nowadays, whey proteins and their derivatives are widely used in the food industry due to the excellent functional and nutritive properties adding to the commercial value of the processed foods [8]. The biological components of whey proteins, including β-lactoglobulin, α-lactalbumin, lactoferrin, lactoperoxidase, immunoglobulins and glycomacropeptides, demonstrate a wide range of immune enhancing properties, and act as antioxidant, antihypertensive, antitumer, antiviral, antimicrobial and chelating agent. They also improve muscle strength and body composition and prevent cardiovascular, cancer diseases and osteoporosis [9].

In spite of their high biological properties, native whey proteins are not hydrolyzed easily by means of digestion enzymes as pepsin and trypsin, due to disulfide bonds in the protein molecules. The poor digestibility of whey proteins is considered to be the reason for their allergenicity [10]. Therefore, modification of whey proteins to enhance or alter their biological and functional properties may increase its applications. Whey protein modification can be accomplished by chemical, enzymatic, or physical techniques [11,12]. Acetylation, succinylation, esterification, amidation, phosphorylation, and thiolation are chemical modifications that induce significant alterations of the structure and functional behavior of whey proteins.

Relatively small alterations of structure, brought about through chemical derivatization, often can be reflected in significant changes of physical and biological properties [13,14].

Many studies concerned with the antiviral activity of native and modified whey proteins in human [15,16]. Other studies focused on the use of milk or milk components to control plant viruses [17]. Therefore the objective of this work was to find and study possible antiviral compounds that would provide effective disease control under practical conditions, while also minimizing environmental impacts using native and modified whey proteins fractions (α-lactalbumin, β-lactoglobuline and lactoferrine) to control TYLCV.

## Materials and methods

### Materials

Healthy tomato, *Lycopersicon esculentum *Mill (Castlerock) seedlings and the severe strain of TYLCV-Is *Tomato yellow leaf curl virus-Israel *(TYLCV-Is [Sever]) [18] were obtained from Virus and Mycoplasma Department, Plant Pathology Research Institute, Agriculture Research Center, Giza - Egypt [19-21]. α-lactalbumin (97.46% protein), β-lactoglobulin (97.8% protein) were kindly obtained from Davisco food international (USA) and lactoferrine (95% protein) were kindly obtained from Armor Proteins (France). All other chemicals used in this study were of analytical grade.

### Methods

#### 1-Protein Esterification

The procedure of [12] was used for esterification of whey proteins fractions using >99.5% methyl alcohol, at 4°C for 10 h. as follows:

Native whey proteins fractions were dispersed (5%, w/v) in methyl alcohol 99.5%. Amounts of hydrochloric acid equivalent to 50 molar ratio of acidity (MR, mole acid/mole carboxyl group) were added drop-wise at the start of the reaction time. All the reaction mixtures were kept at 4°C under continuous stirring. At the end of the reaction (6 h), the samples were centrifuged at 10000 g for 10 min. The resulting supernatant was discarded and the residue was dispersed in a volume of alcohol (99.7% ethanol) equal to that of the discarded supernatant, and well mixed before re-centrifuging at the same conditions. This washing step was repeated three times. The final precipitate was dissolved in an appropriate amount of distilled water then submitted to freeze-drying. The lyophilized samples were kept at -20°C until analysis. The color reaction using hydroxylamine hydrochloride was used according to [22] to quantify the extent of esterification of proteins.

### 2-Experimental

#### Agro-Infiltration with TYLCV-IS infectious clone

Tomato plants previously transformed using optimized *Agrobacerium-Mediated protocol *[19] were agro-infiltrated with the infectious clone of *TYLCV*-IS using the syringe spotted technique (SST) [19-21].

### Treatments

Tomato plants were planted under green house conditions taking into consideration all the environmental requirements conditions of irrigation, fertilization....etc. Plants were then transferred to large coercive after 20 days from planting (5 plants for each treatment). They were submitted to virus infection after 7-10 days from transferring using Agro-Infiltration with *TYLCV*-IS infectious clone. After 10 - 20 days from infection, each plant was sprayed using 20 ml of the native and chemically modified whey proteins fraction at concentration of 1 mg/ml. Leaves were collected from new growth produced after inoculation before treatment, 7 and 15 days after treatment in which total nucleic acids and molecular hybridization analysis were carried out.

### 3-Analytical

#### Detection and quantification of viral DNA

Viral DNA was extracted from tomato tissues using the modified Dellaporta extraction method [23,24].

#### Antiviral activity of modified whey proteins fractions

Antiviral activity was assessed on TYLCV particles replicated in plant tissue, using DNA non-radioactive hybridization [see Additional file 1 for data] to detect the presence and the absence of TYLCV in the treated plants using DNA sequence according to [19-21,24].

The dried DNA pellets were resuspended in 50 μl of TE-RNase buffer (Tris EDTA-RNase buffer) and 5 μl of each sample were dot onto the positively charged nylon membrane. The hybridization experiments were curried out using Gene Images AlkPhos and Chemiluminescent Detection System signal generation and detection with CDP-Star (Amersham, Biosciences, UK Limited) as described by [25-27].

## Results

### Extent of esterification

The whey proteins fractions α-lactalbumin, β-lactoglobulin and lactoferrine were modified at the extent of 68%, 100% and 100% respectively which indicate less esterification susceptibility of α-lactalbumin as compared to both of β-lactoglobulin and lactoferrin. The observed extents of such esterification are in accordance with [12].

### Evaluation of TYLCV infection

Results obtained from PCR carried out on samples taken 10-15 days after infection using two TYLCV specific Primers, TYv 2337, (5'-ACG TAG GTC TTG ACA TCT GTT GAG CTC-'3) and TYc138 (5'-AAG TGG GTC CCA CAT ATT GCA AGA C-'3) [20] indicated that the plants were completely infected by the virus. Infected plants are stunted or dwarfed since only new growth produced after infection is reduced in size. Leaflets are rolled upwards and inwards and leaves are often bent downwards and are stiff, thicker than normal have a leathery texture, show interveinal chlorosis and are wrinkled. Young leaves are slightly chlorotic (yellowish).

### Antiviral activity of whey proteins fractions against TYLCV

#### 1-Antiviral activity of α-Lactalbumin (ALA)

Data presented in Fig. 1(A) &1(B) shows that the virus replication was completely inhibited after 15 days using native ALA (Fig. 1A). In contrast, modified form of ALA (68% methylation extent) gave the same antiviral action such as the native protein after 7 days of application (Fig. 1B).

**Figure 1:** **Antiviral activity of α-Lactalbumin (ALA)**. Antiviral activity of α-lactalbumin (ALA) on infected tomato plants treated with: A) native α-Lactalbumin, B) modified α-Lactalbumin (5 plants for each treatment). 1) Before treatment (zero time), 2) 7 days after treatment, 3) 15 days treatment. 4) Positive control (without treatment), 5) negative control (Healthy plants), 6) infected plants sprayed with water.

#### 2-Antiviral activity of β-lactoglobulin (BLG)

As shown in Fig. 2(A) &2(B), the native and modified forms of BLG had a little antiviral activity.

**Figure 2:** **Antiviral activity of β-lactoglobulin (BLG)**. Antiviral activity of β-lactoglobulin ((BLG) on infected tomato plants treated with: A) native β-lactoglobulin, B) modified β-lactoglobulin (5 plants for each treatment). 1) Before treatment (zero time), 2) 7 days after treatment, 3) 15 days treatment. 4) Positive control (without treatment), 5) negative control (Healthy plants), 6) infected plants sprayed with water.

#### 3-Antiviral activity of Lactoferrin

Fig. 3(A) &3(B) shows that lactoferrin inhibits the virus replication completely in infected plants either the native or the modified form even after 7 days from spraying.

**Figure 3:** **Antiviral activity of Lactoferrin**. Antiviral activity of lactoferrin on infected tomato plants treated with: A) native lactoferrin, B) modified lactoferrin (5 plants for each treatment). 1) Before treatment (zero time), 2) 7 days after treatment, 3) 15 days treatment. 4) Positive control (without treatment), 5) negative control (Healthy plants), 6) infected plants sprayed with water.

## Discussion

Esterification is an important and easy tool of protein modification. Esterification blocks free carboxyl groups raising thus the net positive charge and rendering more basic the modified protein. It has been recently reported that increased basicity of dairy proteins after their esterification endow them with DNA-binding properties [12,14,28].

Early studies led to several hypotheses about milk's mode of action. The first one was in the 1930s suggested that milk inhibited infection by somehow reducing the plant's susceptibility to the virus [7]. The second one in the 1940s suggested that the milk "inactivated" the virus by forming a loose "molecular union" which, if broken, results in re-activation of the virus. That is, the inhibiting effects were reversible and the effect was on the virus and not the plant. The studies of an Australian scientist in the 1950s supported the earlier hypothesis that milk contains a substance that inhibits virus infection due to its effect on the plant, by supposedly inducing some type of resistance. It was also found that the inhibitory effects were restricted only in the treated part of the plant. Furthermore, investigations suggested that the active substance in the milk was a protein. The conclusion that the active substance is a protein component or number of such components is supported by recent work carried out by USDA scientists. But the answer to how exactly milk inhibits or reduces virus infection is still unknown [6,7].

Milk is rather heterogeneous suspension of oil (butter-fat), protein (cassein), sugar (lactose) and a multitude of possibly bioactive trace ingredients, including minerals, enzymes and vitamins. Possible modes of action of milk-based sprays were provided by [29]. These include an increase in the pH of the leaf surface [30], the establishment of a protective barrier, the establishment of possibly antagonistic organisms [31,32] the direct induction of systemic resistance [33] and/or the production of biocidal compounds [34]. All of the above processes will probably be highly dependent on the environmental conditions and the timing of the epidemic with respect to the phenology of the crop.

Milk contains several salts and amino-acids. These substances have been shown to be effective in controlling powdery mildew and other diseases [31-33,35-37].

The obtained results reveal that the antiviral activity of lactoferrin (either native or purified form) is greater than α-lactalbumin or β-lactoglobulin.

Milk whey proteins acquire net positive charges after esterification with methanol or ethanol enabling them to interact with negatively charged macromolecules such as nucleic acids or some proteins [12]. Consequently, these basic proteins may interact with viral DNA or RNA. Esterification not only increases the gross positive charge of the protein but also its hydrophobicity by grafting hydrophobic methyl or ethyl groups on the carboxyl groups of aspartyl and glutamyl residues. Enhanced hydrophobicity may also promote hydrophobic interactions with the hydrophobic binding sites formed by viral capsid proteins. Some antiviral inhibitory effects were already explained by the entry of hydrophobic inhibitory molecules in the hydrophobic binding cavities on the viral surface [38-40].

The interaction of antiviral proteins such as LF with receptors on cell surface and/or with viral envelope proteins is critical to blocking viral entry to target cells. The charge on the antiviral protein plays an indispensable role in this interaction. Chemical modifications lead to changes in the charges on milk proteins which can enhance their antiviral properties [41,42].

The results indicate that the inhibition of TYLCV may be related to the degree of cationisation of esterified whey proteins as well as to the size of the backbone protein which could be due to:1) Saturating binding to viral DNA by purely coulombic interactions, inhibiting its replication and transcription; 2) Hydrophobic interactions with viral capsid proteins; 3) Perturbation of viral DNA-protein interactions, hence inhibition of the translation of viral proteins; 4) Interference with/saturation of viral entry sites on the cellular membranes.

Many researchers recommend the use of milk to reduce the spread of virus particles between plants. Techniques using milk are frequently used in nurseries to stop the spread of virus between susceptible hosts when people touch the plant, during pruning. They reported milk proteins inactivated the capsid protein of the virus. Milk is not a potential environmental or food contaminant; consequently it can be used in organic agriculture.

Also, the data of [43-45] indicated that whey was effectively used to control powdery mildew in cucumber and zucchini and they recommended further studies to optimize the concentration and timing of whey applications for mildew management in commercial crops.

The antiviral effect of the used whey protein fractions can be arranged in descending order as follows: lactoferrin (native or modified form) > native α-lactalbumine > modified β-lactoglobulin > modified α-lactalbumin = native β-lactoglobulin. More studies are needed to improve the antiviral activity of both of α-lactalbumin and β-lactoglobulin.

In future experiments, we will examine combined regimen of alternating milk-based and chemical sprays and also using different concentration of whey, whey protein fractions and skim milk. These strategies may provide adequate protection against this disease, while reducing the chemical load on the environment and forestalling the development of resistant strains.

Finally the use of alternative "green" methods would have its advantage in the market, as many consumers are ready to pay more for pesticide-free products. This point could be of enough interest to justify the present work.

## Competing interests

The authors declare that they have no competing interests.

## Authors' contributions

AMA conceived the research, performed the experiments, and wrote the manuscript; SHT developed the conceptual aspects of the work and edited the manuscript; MIS conceived of the study, and participated in its design and coordination; AZA participated in the design of the study; MMA conceived the research, performed the experiments, and edited the manuscript; AAR carried out the molecular genetic studies. All authors read and approved the final manuscript.

## Supplementary Material

Additional file 1 **Antiviral activity of modified whey proteins fractions**. The data provided represent the DNA sequence used in DNA non-radioactive hybridization. Click here for file

## References

[B1] Abdel-SalamAMIsolation and characterization of a whitefly-transmitted geminivirus associated with the leaf curl and mosaic symptoms on cotton inEgypt Arab J Biotech19992193218

[B2] Abdel-SalamAMEI-ShazlyAMThouvenelJCBiological and biochemical studies on hollyhock leaf crumple virus (HLCrV): A newly discovered whitefly-transmitted geminivirusArab J Biotech19981418

[B3] Abdel-SalamAMSolimanZDEL-BannaMOCharacterization of a geminivirus infection tomato plant in Egypt3rd International Geminivirus symposium at John Innes Centre, Norwich, UK on 2001, 24-28, July

[B4] FadlGMBurgstallerHReduction of tomato leaf curl virus in Sudan through variety selection and insecticide applicationActa Horticulture1984190159164

[B5] FanigliuloAComesSCrescenziAMomolMTOlsonSMSacchettiMFerraraLCaligiuriGIntegrated management of tomato yellow leaf curl in protected tomato crops in southern ItalyActa Horticulture (ISHS)2009808393396

[B6] College of agriculture of scienceCharles W AverrePlant pathology extension (2000). Virus Diseases of Greenhouse Tomato and Their Management. Vegetable Disease Information Note 15 (VDIN-0015)Research Plant PathologistExtension Plant pathologist Guy V. Goodinghttp://www.ces.ncsu.edu/depts/pp/notes/oldnotes/vg15

[B7] GillianFMilk as a Management Tool for Virus Diseases2005http://www.omafra.gov.on.ca/english/crops/hort/news/grower/2005/11gn05a1.htm16287997

[B8] JovanovićSMiroljubBOgnjenMWhey proteins-Properties and Possibility of ApplicationMljekarstvo200555215233

[B9] MarshallKTherapeutic applications of whey proteinAlternative Medicine Review2004913615615253675

[B10] SchmidtDGMeijerRJSlangenCJvan BeresteijnECRaising the pH of the pepsin-catalysed hydrolysis of bovine whey proteins increases the antigenicity of the hydrolysatesClinical and Experimental Allergy1995251007101710.1111/j.1365-2222.1995.tb00404.x8556555

[B11] KananenASavolainenJMaK kinenJPerttilaKUMyllykoskiLPihlanto-LeppaKAInfluence of chemical modification of whey protein conformation on hydrolysis with pepsin and trypsinInternational Dairy J20001069169710.1016/S0958-6946(00)00094-7

[B12] SitohyMChobertJMHaertléTSimplified short-time method for the esterification of milk proteinsMilchwissenschaft200156127131

[B13] RyanDSFeeney RE, Whitaker JRDeterminants of the functional properties of proteins and protein derivatives in foods. in Food proteinsImprovement through chemical and enzymatic modification1977Washington, DC67

[B14] SitohyMMicheleDMarieNBesseBBillaudelSHaertleTChobertJMThe effect of bovine whey proteins on the ability of poliovirus and Coxsackie virus to infect Vero cell culturesInternational Dairy J20081865866810.1016/j.idairyj.2007.11.023

[B15] ChobertJMSitohyMBillaudelSMicheleDHaertleTAnticytomegaloviral activity of esterified milk proteins and L-PolylysinesJ Mol Microbiol Biotechnol20071325525810.1159/00010475517827977

[B16] PanYLeeAWanJCoventryMJMichalskWPShiellBRoginskiHAntiviral properties of milk proteins and peptides (A Review)International Dairy J2006161252126110.1016/j.idairyj.2006.06.010

[B17] LiakotMAAsadDPramanikBkAshrafuzzamanMManagement of leaf curl disease of Tomato. PakistanJ Biolo Science2001415121514

[B18] NavotNPicherskyEZeidanMZamirDCzosnekHTomato yellow leaf curl virus: a whitefly-transmitted geminivirus with a single genomic componentVirology199118515116110.1016/0042-6822(91)90763-21926771

[B19] AhmedFHGhandiHAnfokaGDhiaSHTransformation of tomato with TYLCV gene silencing construct using optimizedAgrobacerium-Mediated protocol Biotechnology200873537543

[B20] AnfokaGAbharyMHaj AhmadFHusseinAFRezkAAkadFAbou-JawdahYLapidotMVidavskiFNakhlaMKSobhHAtamianHCohenLSobolIMazyadHMaxwellDPCzosnekHSurvey of tomato yellow leaf curl disease-associated viruses in the eastern mediterranean basinJournal of Plant Pathology2008902311320

[B21] RezkAAInduction of TYLCV resistant plants through tools of molecular biologyPhD thesis2006Agricultural Science, Department of Plant Pathology, Faculty of Agriculture, Cairo University

[B22] Bertrand-HarbCChobertJMDufourEHaertleTEsterification of food proteins: Characterization of the derivatives by a colorimetric method and by electrophoresisSciences des Aliments199111641652

[B23] DellaportaSLWoodJHicksJBA plant DNA minipreparation: version IIPlant Mol Biol Rep19831192110.1007/BF02712670

[B24] RezkAANakhlaMKAbo El-AbbasFMEl-HammadyMHMazyadHMMaxwellDPMolecular methods for detection of banana bunchy top virus (BBTV) from banana tissues and viruliferous banana aphidAPS annual meeting. July 2002, Wisconsin, USA

[B25] AbharyMKPathogen derived resistance for controlling tomato yellow leaf curl virus (TYLCV)MSc Thesis2003Al-Balqa Applied Univ. Fac. Agric. technology, Dept. Biotechnology, Jordan

[B26] JohansenLKCarringtonJCSilencing on the spot. Induction and supression of RNA silencing in the Agrobacterium-mediated transient expression systemPlant Physiol200112693093810.1104/pp.126.3.93011457942PMC1540124

[B27] PotterJLNakhlaMKMejíaMMaxwellDPPCR and hybridization methods for specific detection of bean-infecting begomoviruses in the Americas and CaribbeanPlant Dis2003871205121210.1094/PDIS.2003.87.10.120530812724

[B28] SitohyMChobertJMThomasHEsterified whey proteins can protect Lactococcus lactis against bacteriophage infection. Comparison with the effect of native basic proteins and L-polylysinesJournal of agricultural and food chemistry2005533727373410.1021/jf048629z15853427

[B29] BettiolWEffectiveness of cow's milk against zucchini squash powdery mildew (*Sphaerotheca fuliginea*) in greenhouse conditionsCrop Protection19991848949210.1016/S0261-2194(99)00046-0

[B30] ZivOZitterTAEffects of bicarbonates and film-forming polymers on cucurbit foliar diseasesPlant Disease1992265513517

[B31] McGrathMTShishkoffNEvaluation of biocompatible materials for managing cucurbit powdery mildewCrop Protection19991847147810.1016/S0261-2194(99)00048-4

[B32] MucharromahEKucJOxalate and phosphates induce systemic resistance against diseases caused by fungi, bacteria and viruses in cucumberCrop Protection199110326527010.1016/0261-2194(91)90004-B

[B33] ReuveniMAgapovVReuveniRInduction of systemic resistance to powdery mildew and growth increase in cucumber by phosphatesBiological Agriculture and Horticulture199394305315

[B34] TzengDDSDeVayJEBiocidal activity of mixtures of methionine and riboflavin against plant pathogenic fungi and bacteria and possible mode of actionMycologia19898140441210.2307/3760078

[B35] PasiniCD'AquilaFCurirPGullinoMLEffectiveness of antifungal compounds against rose powdery mildew (Sphaerotheca pannosa var. rosae) in glasshousesCrop Protection199716325125610.1016/S0261-2194(96)00095-6

[B36] ReuveniMAgapovVReuveniRSuppression of cucumber powdery mildew (Sphaerotheca fuliginea) by foliar sprays of phosphate and potassium saltsPlant Pathology1995441313910.1111/j.1365-3059.1995.tb02713.x

[B37] TitonePMigheliQAcutisMGaribaldiAIl fosfato monopotassico nella lota al mal bianco dello zucchinoColture Protette199847379

[B38] CoxSBuontempoPJWright-MinogueJde MartinoJLSkeltonAMFerrariEAntipicornavirus activity of SCH47802 and analogues: In vitro and in vivo studiesAntiviral Research199632717910.1016/0166-3542(95)00979-58891166

[B39] O'ConnellJFAlbinRBlumDGrintPSchwartzJRotbart HADevelopment of antiviral agents for picornavirus infectionsHuman enterovirus infections1995Washington, DC, USA: ASM Press419434

[B40] SkeltonAMFerrariEAntipicornavirus activity of SCH47802 and analogues: In vitro and in vivo studiesAntiviral Research199632717910.1016/0166-3542(95)00979-58891166

[B41] SwartPJHarmsenMCKuipersMEVan DijkAAStrateBW Van derVan BerkelPHCharge modification of plasma and milk proteins results in antiviral active compoundsJournal of Peptide Science1999556357610.1002/(SICI)1099-1387(199912)5:12<563::AID-PSC226>3.0.CO;2-310628656

[B42] WaartsBAnekeOJSmitJMKimataKBittmanRMeijerDKFAntiviral activity of human lactoferrin: Inhibition of alphavirus interaction with heparan sulfateVirology200533328429210.1016/j.virol.2005.01.01015721362

[B43] BettiolWHarllenSAReisRCEffectiveness of whey against zucchini squash and cucumber powdery mildewScientia Horticulturae2008117828410.1016/j.scienta.2008.03.010

[B44] CrispPScottESWicksTJEvaluation of biological and novel control of grapevine powdery mildewProceedings of the 15th Australasian Plant Pathology Society Conference Handbook, Geelong, Australia200585

[B45] CrispPWicksTJTroupGScottESMode of action of milk and whey in the control of grapevine powdery mildewAust Plant Pathol20063548749310.1071/AP06052

